# Ensemble learning for multi-class COVID-19 detection from big data

**DOI:** 10.1371/journal.pone.0292587

**Published:** 2023-10-11

**Authors:** Sarah Kaleem, Adnan Sohail, Muhammad Usman Tariq, Muhammad Babar, Basit Qureshi

**Affiliations:** 1 Department of Computing and Technology, Iqra University, Islamabad, Pakistan; 2 Iqra University, Islamabad, Pakistan; 3 Abu Dhabi University, Abu Dhabi, UAE; 4 Universiti Tun Hussein Onn Malaysia (UTHM), Parit Raja, Malaysia; 5 Robotics and Internet of Things Lab, Prince Sultan University, Riyadh, Saudi Arabia; 6 College of Computer and Information Sciences, Prince Sultan University, Riyadh, Saudi Arabia; Menoufia University, EGYPT

## Abstract

Coronavirus disease (COVID-19), which has caused a global pandemic, continues to have severe effects on human lives worldwide. Characterized by symptoms similar to pneumonia, its rapid spread requires innovative strategies for its early detection and management. In response to this crisis, data science and machine learning (ML) offer crucial solutions to complex problems, including those posed by COVID-19. One cost-effective approach to detect the disease is the use of chest X-rays, which is a common initial testing method. Although existing techniques are useful for detecting COVID-19 using X-rays, there is a need for further improvement in efficiency, particularly in terms of training and execution time. This article introduces an advanced architecture that leverages an ensemble learning technique for COVID-19 detection from chest X-ray images. Using a parallel and distributed framework, the proposed model integrates ensemble learning with big data analytics to facilitate parallel processing. This approach aims to enhance both execution and training times, ensuring a more effective detection process. The model’s efficacy was validated through a comprehensive analysis of predicted and actual values, and its performance was meticulously evaluated for accuracy, precision, recall, and F-measure, and compared to state-of-the-art models. The work presented here not only contributes to the ongoing fight against COVID-19 but also showcases the wider applicability and potential of ensemble learning techniques in healthcare.

## 1 Introduction

COVID-19 (Novel Coronavirus) was found in December 2019 in a cluster of unknown pneumonia patients [1–3]. COVID-19 has been announced as an international concern and community health emergency by WHO (World Health Organization) [4]. The WHO emergency panel has indicated that the blowout of COVID-19 could be broken up by rapid discovery, segregation, early cure, and execution of a vigorous method to trace interactions [5]. Covid-19 has a significant impact on human lives across the globe. The world has responded generously after the COVID-19 outburst. The COVID-19 outbreak has led the leading agencies to fund research projects to overcome the current crisis. These agencies include the EU (European Union) mobilizing a €10 million fund (research-oriented) for more proficient clinical administration of COVID-19 confirmed cases, US-based companies have tossed testing kits for research [6], an investment of £20 million done by the UK government for developing a vaccine [7]. The countries have responded strictly to this outbreak, the new coronavirus COVID-19 [8]. The number of confirmed cases increased rapidly in China and across the globe, with infected patients having no link with close contact with the infected person.

By contrast, Data Science and Machine Learning practices have solved numerous long-standing multifarious problems [9,10]. There is no prospect that Data Science and Machine Learning methods will instantaneously resolve COVID-19. These techniques can offer an intense consideration of COVID-19 and its societal effects. An extra vigilant investigation based on existing data and expressive predictions could be valuable for decision making and future policies. In the context of COVID-19, people have started working on predicting the growth of COVID-19 patients using the concepts of Data Science and Machine Learning. Most countries have controlled COVID-19 to a large extent because they use Big Data and Machine Learning to try the highest technology epidemic control ever in the history of the world. They have taken significant safety measures to control crises using big-data analytics and Machine Learning. They are accumulating massive amounts of Big Data about their people and using it innovatively (AI and Machine Learning) to address current disasters. Machine Learning analytical approaches were utilized for the final size prediction. Similarly, models based on EIR (Exposed-Infected-Recovered (EIR), SIR (Susceptible-Infected-Recovered), and Susceptible-Infected-Recovered-Deceased (SIRD) are also used to predict the growth of patients with COVID-19 [11]. It is necessary to predict the development of COVID-19 to control future panic worldwide.

The application of machine learning techniques to study and management of the Corona Virus has significantly contributed to health safety measures, enabling rapid improvement in patient care [12]. Among the most significant elements is identifying disease-outbreak viruses by predicting whether SARS-CoV-2 can transmit disease to humans. SARS-CoV-2 is spread by infected individuals with drops of saliva, the common cold, and sniffles. Most citizens diseased with SARS-Cov-2 have mild lung disease, but those with medical conditions such as vascular disease, obesity, severe pulmonary disease, or leukemia are more likely to develop a medical condition. People who are older than 65 years and have medical issues are at a higher risk of contracting this disease. Currently, no vaccines or therapies are available for SARS-CoV-2. The accurate detection of COVID-19 with efficient training and execution time still needs to be included. Therefore, Machine Learning and Data Science techniques can offer a profound understanding and analysis of COVID-19. It can also provide information on the impact and behavior of the COVID-19 crisis on societies worldwide. At this stage of the COVID-19 outbreak, an extra vigilant investigation based on available existing data and expressive Machine Learning techniques could be valuable for decision-making and future policy setting. Machine learning and artificial intelligence (AI) solutions are extremely useful for resolving these issues.

The diagnostic criteria were based on history and clinical indicators. The data suggested the severity of COVID-19 deaths in the region and preparing health care for timely actions. The comparison shows that COVID-19 deaths follow the Boltzmann function [13]. The prospective number of deaths was calculated by applying Richard function-based regression analysis, which simulated the accumulative confirmed cases of SARS 2003 in different regions to verify the estimation. Another study on COVID-19 prediction and analysis was conducted using artificial intelligence. The correlation between attributes and labels was evaluated as two essential indicators for ranking the characteristics of medical records.

The capability to promptly detect and quarantine diseased persons is one of the most necessary procedures for eradicating COVID-19. The capability to detect diseased persons timely and place them in quarantine is one of the most necessary procedures for eradicating COVID-19. One of the most practical ways to analyze COVID-19 patients was to use radiology and radiography images to diagnose this condition. Chest radiography is the initial and most economical test procedure. Therefore, there is a need to recognize the presence of COVID-19 in patients using chest X-rays, which could benefit individuals and society. The existing COVID-detecting techniques from X-rays can be more efficient in terms of training and execution times. Using a Machine Learning technique, this article proposes an architecture for detecting COVID-19 from chest X-ray images. The proposed model uses a parallel and distributed framework to perform parallel processing, whereas it uses a parallel and distributed framework to perform parallel processing. The ensemble learning method for machine learning is equipped with the proposed architecture. The models were trained in parallel to improve the execution and training time of the detection process.

## 2 Related work

Detection of a virus involves various methods, of which testing is the only one. The emergence of AI and ML for handling previous pandemics has opened new avenues for researchers in the battle against COVID-19. These technologies offer a new perspective that transcends traditional approaches. Specifically, the application of AI and machine learning has become crucial in areas related to SARS-CoV-2, including pandemic screening, prediction, forecasting, contact tracking, and development of treatment strategies. By integrating these modern techniques, the healthcare community is enhancing its ability to understand and control the spread of the virus [14].

Machine Learning has garnered widespread recognition across multiple domains due to its ability to convert raw data into valuable insights, predictions, and decision-making tools. This versatility and compatibility across various fields have established Machine Learning as a pivotal technology in contemporary research and development [10].

Deep learning techniques have been successfully utilized to model groundwater storage changes, providing a data-driven approach to understanding subsurface water dynamics, which is a crucial component in water resource management [15]. CDLSTM is a new model for forecasting climate change was developed by incorporating Convolutional LSTM networks [16]. This approach has allowed researchers to make more accurate predictions of climate change patterns and to better prepare for the challenges posed by these changes [17]. The incorporation of AI and ML into environmental research has facilitated the examination of intricate interactions within ecosystems [18]. This has resulted in new perspectives on environmental conservation and management approaches. ML algorithms have been employed for classifying images captured by nanosatellites, such as PlanetScope, which has opened up new possibilities for remote sensing and space exploration [17]. The use of Convolutional Neural Networks (CNN) in conjunction with Unmanned Aerial Vehicles (UAVs) has revolutionized weed detection in agriculture. Automation leads to more efficient and sustainable farming practices [19].

Employing deep learning algorithms for the classification of forest areas through UAV imagery has proven to be a valuable advancement for forestry management and conservation efforts [19]. The emergence of advanced deep neural network models, such as DBOTPM, has significantly strengthened cybersecurity efforts by facilitating the timely identification and containment of botnet attacks. A new model named SMOTEDNN has been introduced for air pollution forecasting and Air Quality Index (AQI) classification, which helps in pollution control and making informed decisions related to public health [17].

These diverse applications of ML not only demonstrate its broad utility but also provide a substantial justification for its implementation in the present work. By showcasing the success of ML across different fields, it sets the stage for its application in detecting COVID-19 from chest X-ray images, further promoting the idea that ML techniques can bring transformative changes and innovations to even more sectors in the future [19].

## 3 Applications of machine learning in healthcare

The impact of ML and Deep Learning on healthcare is evident across multiple medical specialties, transforming the way diseases are identified, diagnosed, and treated. These advancements are improving patient care, increasing efficiency, and providing personalized therapeutic solutions. Some notable examples of their contributions are as follows:

Deep convolutional neural networks (CNNs) are the driving force behind the revolutionary DCNNBT model for brain tumor classification [20]. This method enables swift and accurate diagnosis, simplifying the decision-making process for treatment by processing intricate imaging data. The model provides healthcare professionals with unparalleled insights into tumor types and stages, ultimately guiding targeted therapeutic interventions. The shortage of high-quality medical images presents a significant obstacle to training strong ML models [21]. This groundbreaking method employs data augmentation techniques to artificially increase the dataset and applies transfer learning to utilize pre-trained models. This combination overcomes the limitations of data availability and enables more efficient brain tumor identification. This approach demonstrates the versatility of ML in addressing the unique challenges of healthcare, thereby making diagnoses more dependable and accessible [22].

Magnetic Resonance (MR) imaging of the brain plays a vital role in neurology and neurosurgery. By adopting the U-Net architecture, the segmentation of MR brain images was optimized, leading to increased precision in identifying the brain structures [23]. This enhanced accuracy in delineating tumors, blood vessels, and other anatomical features not only enhances diagnostic capability but also aids surgical planning. This technological advancement represents a fusion of cutting-edge technology and medical expertise, heralding a new era of neurological care. Personalized medicine, a rapidly growing field in oncology, aims to tailor treatments to individual patient characteristics by predicting the responsiveness of cancer cells to antiangiogenic inhibitors, a class of drugs that impede blood vessel formation in tumors [24]. This approach provides oncologists with informed treatment decisions, offers insights into the likely success of these inhibitors, and promises more targeted and effective cancer treatments [25].

The applications outlined above demonstrate a powerful combination of machine learning and medical sciences. They showcase not only technological advancements but also a shift towards a more responsive and personalized healthcare system. These models offer exciting insights into the future of medical practice, where machine learning algorithms continuously learn and adapt to the evolving needs and complexities of the field, providing clinicians with intelligent tools that enhance decision-making and improve patient outcomes [26].

The recognition of COVID-19 patients is a complex task and requires multiple test procedures that are costly and time-consuming [27]. Chest radiography is the initial and most economical test procedure for these tests. Therefore, there is a need to recognize the presence of COVID-19 in patients through chest X-rays, which could benefit individuals and society [28]. Since its outbreak, it has spread rapidly across the country with conditions such as pneumonia. This has triggered an internal threat to become a global pandemic. Two other coronaviruses have occurred since 2002, which caused similar acute respiratory syndromes to spread to 37 countries. It has been observed that diseases should have an early prediction of an outbreak by formulating a dynamic system to predict the course of the disease and to devise different management strategies. These issues may arise from a late forecast that can cause problems in the timely prediction of the epidemic, which can cause more harm than benefit. Researchers have focused on developing a simple approach for a prediction that can analyze the decrease in contact rates in time according to the response to the disease outbreak.

CT and X-ray images identify and localize SARS-CoV-2 contaminated regions [29]. While there is no specific antiviral treatment or cure for SARS-CoV-2, the virus that causes COVID-19, several medical interventions and supportive care measures are available to manage symptoms. Machine learning models have been utilized to further contribute to the care and understanding of the disease, such as recognizing SARS-CoV-2 patients from heart video sequences. In this innovative approach, the texture function is generated using the FFT spectrum, and the image is analyzed using a regular clustering algorithm [30]. Individuals diseased with the coronavirus have severe breathing problems requiring ICU medication. SARS-CoV-2 has a low mortality rate of less than 3%; however, its extreme death rate is high. The training and research datasets included various cases of SARS-CoV-2-affected individuals. Another method was proposed to identify SARS-CoV-2 using a deep-running method using high-resolution photographs. The matrix system employs a dense model to identify the Y and Z frames. The SVM and resnet50 classification models have been proposed [31]. This is a DL-enabled system for identifying SARS-CoV-2 from chest X-rays [31]. SARS-CoV-2 was detected using ResNet18, ResNet50, SqueezeNet, and DenseNet-121. They utilized a dataset of 5000 images [32]. The proposed system needs to improve the training and execution times. Thus, the accuracy could have improved. A group of researchers have utilized a deep learning method to classify SARS-CoV-2 from CXR images, where the CXR dataset was used from a Northern Italy hospital [33]. The planned DL method highlighted the effectiveness of the COVID-Net architecture for training.

Another DL model based on metaheuristics is presented using chest images to detect COVID. This method was used to classify the input images, along with feature extraction. An optimized AlexNet design was utilized for the classification [34,35]. This model classifies chest images into various categories including other diseases. The accuracy is compromised owing to multi-classification. The training and execution times were also high. A Deep Convolutional Neural Network (DCNN)-enabled model was proposed to recognize COVID-19 cases. The proposed method uses several cutting-edge CNN models, including DeneNet201, Resnet50V2, and Inceptionv3 [36]. A novel attention-oriented DL technique using VGG-16 was proposed to capture the spatial relationship between ROIs in CXR images [37]. To detect pneumonia in chest images, a hybrid DL technique utilizes various mechanisms, including DenseNet121, Inception-ResNet-V2, Resnet50, Xception, VGG16, VGG19, and InceptionV3 [38]. A hybrid ensemble model classifier was used to distinguish COVID-19 from common viral pneumonia based on chest X-ray [39]. A concatenated neural network was used to classify X-ray images by merging many features with several robust networks. It has high accuracy, but the execution and training times also increase [40]. A deep learning multi-classification model was developed using an amalgamation of chest X-ray and CT images to identify COVID-19, lung cancer, and pneumonia [41].

The susceptible-expose-infectious-recovered (SEIR) model is based on the assumption of uncovered-infected individuals [33]. The actual cases were far more than the reported cases, which can be inferred as an epidemic that could have spread due to exposed individuals who were incubated. The SIR model was used to identify the number of infected, susceptible, and removed persons in mainland China who were infected with COVID-19. The number of victims in an area was predicted to analyze the initial phases of the epidemic, which can help plan future outbreaks [42]. The susceptible-infected-recovered-dead SRID (model was used to analyze the values according to confirmed cases. A common question about the epidemic still needs to be added to the final size and peak time. Various models have been used, such as analytical, stochastic, phenomenological, and EIR, to predict the infection size and peak time. Logistic model and regression analysis were used to estimate population dynamics per capita. Screening of 2799 patients’ records was performed to evaluate the criticality of infection based on the clinical features: a prognostic model (ML-based), which estimated the mean age of 375 patients. The model was further analyzed for lactic dehydrogenase, lymphocytes, and high sensitivity [43]. Privacy-preserving methods for medical record security have also been proposed [44,45]. It is depicted from the current literature in the context of COVID-19 and Machine Learning that accurate detection of COVID-19 for efficient training and execution times is still missing. It is depicted from the current literature in the context of COVID-19 and Machine Learning that the accurate detection of COVID-19 for efficient training time and execution time is still missing.

## 4 Material and methods

A detailed description of the proposed method is provided in this section. Fig 1 presents abstract insights into the proposed model. The primary purpose of the proposed model is to detect COVID-19 from chest X-ray images with improved training and execution times with reasonable accuracy. Initially, data preparation was performed, including the application of various pre-processing techniques to the dataset. When using a complex ensemble composed of deep models, such as VGG-16, VGG-19, and ResNet-50, the process of splitting data for training and testing is crucial. Proper data splitting ensures robust evaluation of the model’s performance. The dataset was divided into training and testing sets. The common split ratio was 80% for training and 20% for testing.

**Fig 1:** Workflow of the proposed model.

The data were thoroughly examined to select the responses, features, attributes, and predictors before model development. Subsequently, the model-building process was conducted in a parallel fashion using the optimized parallel and distributed framework. The ensemble learning method was selected to combine the optimal and partial results. This prediction model is preferred because it is widely used and very useful for detection based on the available dataset. In addition, it determines the strength of the detector. This technique is a specific prediction model that investigates the relationship between the independent and dependent variables. The proposed framework includes a dataset and methodology (preprocessing, training model, and validation and classification). The proposed system is illustrated in Fig 2. The proposed model includes two central units: preprocessing and parallel model building.

**Fig 2:** Proposed model.

### 4.1 Preparation and pre-processing

A collection of 6500 chest X-rays were obtained from a public database. Certified radiologists exposed radiology images to the occurrence of COVID-19 [35]. Transfer learning was applied to a subset of 3,500 images, transfer learning was applied. Transfer learning was applied to a subset of 3,500 images from the total collection of 6,500 chest X-rays for several strategic reasons. First, utilizing a subset allowed us to establish a validation set that could be leveraged to fine-tune model parameters without the risk of overfitting. It also facilitates a more balanced representation of the various classes within the dataset, ensuring that the training set has a more uniform distribution. Second, using a subset for transfer learning allows greater computational efficiency. Training on a reduced dataset can often yield comparable performance, while significantly reducing both the training time and computational resources required. This approach often enables iterative experimentation and tuning, leading to a more refined final model. Finally, the use of a subset provided a pragmatic way to assess the effectiveness of transfer learning as compared to training from scratch or using other techniques. By initially applying transfer learning to a subset of the data, the research team could evaluate its impact on model performance and then decide whether to scale the approach to the entire dataset based on the results obtained. This strategic decision-making process enabled the research to be more focused and resource-efficient, while still aiming to achieve robust performance in the detection of COVID-19 from chest X-ray images.

All the X-ray images were initially gathered into a single dataset and then randomly divided into training and testing datasets. Subsequently, they were scaled to a standardized size of 235 × 235 pixels for use in the DL pipeline. The data were combined and gathered into a single dataset using Eq 1.


$$IMG=[IMG_{1},IMG_{2},\ldots IMG_{n}]$$ (1)

Where IMG_i_ is an image with a size of 235 × 235 × 1.

The dataset was split into training and testing datasets, as shown in Eq 2. Subsequently, labels are created for vectors using Eq 3.


$$X_{train},X_{test}=random_{split}(X,n_{train},n_{test})$$ (2)

$$Y_{train}=[Y_{1},Y_{2},\ldots Y_{n_{train}}]$$ (3)

$$Y_{test}=[Y_{n_{train+1}},Y_{n_{train+2}},y_{n}]$$

### 4.2 Model building and processing unit

The pre-processed data were split 75–25 to begin the training phase in a parallel fashion. The use of the Apache Spark parallel and distributed framework in the proposed model was critical for managing a large dataset of 6,500 images. Spark was selected because of its ability to perform efficient parallel processing, which resulted in an improved training time. The distributed nature of Spark enables the system to handle large-scale data with a high computational efficiency. The decision to use Spark was based on its ability to significantly reduce both the training time and computational resources required, making it a suitable choice for handling a 6,500-image dataset. The DL model was trained in parallel to achieve improved training time. The testing part utilized 25% of the image information, whereas the testing part utilized 25% of the image information. Again, 75% of the information was separated to create the same number of validation and training sets.

A random sample of training data was selected for classification. Different standard CNN models, including DenseNet-121, ResNet50, ResNet18, and Squeeze Net, were trained in parallel to detect COVID-19. The input images, with all dimensions and numbers of channels, are expressed in Eq 4. The initial layer of ResNet50 is convolutional, which applies a set of filters to the input image, along with weight and bias.


F1=Conv(InputImage,W1)+b1 (4)

The output was then passed through a series of residual blocks containing two convolutional layers with batch normalization and ReLU activation functions. The output of the last residual block is then passed through a global average pooling layer, as expressed in Eq 5.


F2=ResBlock(F1) (5)

F3=ResBlock(F2) (5.1)

GAP=GlobalAvgPool) (5.2)

FC=FullyConnected(GAP)) (5.3)

Y=Sogtmax(FC)) (5.4)

The X-ray labels were applied with encoding to specify whether the image in the collection had a positive case of COVID-19. The testing dataset was used to tune the classifier that classified the images. The pre-trained models included VGG-16, VGG-19, ResNet, and ImageNet.

The convolutional layers perform operations on the input data, denoted by K. The output of the layer can be represented by Eq 6, where CN(Y_(i,j)) denotes the output at position (i,j) and Z_(i-l,j-m) represents the input data at location (i-l,j-m).


$$CN(Y\_(i,j))=\sum_{x=-a/2}^{a/2}\sum_{l=-n/2}^{n/2}F_{z}(l,m)Z_{i-l,j-m}$$ (6)

Multiple filters, denoted by ft, are utilized to capture a more diverse and rich representation of the input. The filters shown in Eq 7 are applied to the input data within a sliding window of size (n × a), centered at each output position (i,j), and the results are summed to compute the output value at (i,j).


$$FILTERS=F_{Z}(L,M)$$ (7)

After the convolution operation, a rectified linear unit (ReLU) is applied to the output. This can be represented by Eq 8, where RECT(Z) denotes the ReLU output, and max (O, Z) represents the maximum value between 0 (denoted as O) and the input value Z.


$$R_{Z}={M(O,Z)}_{Z}$$ (8)

The ReLU activation function is preferred over other functions such as the sigmoid function because it enables faster convergence during training and overcomes the issue of vanishing gradients by having a linear gradient. Following ReLU, a pooling layer is applied, which can be implemented using various techniques such as average, maximum, and minimum pooling. Among these, the maximum-pooling technique is the most popular. Given a polling filter of size p, the output of the maximum pooling operation is computed using Eq 9, where M(Z_i) represents the output value at positions i and j and max{Z_(i+n,i+m)} denotes the maximum value within the pooling filter centered at (i,j).


$$M(Z_{i})=\max\;\{Z_{i+n,i+m}\}$$ (9)

Various metrics can be employed when evaluating the performance of the machine learning model for identifying COVID-19 from chest X-ray images. Among these, the F-1 score may be a crucial performance metric. Here is an explanation of the metrics, including the formulas, and an explanation of why F-1 is typically used.

Precision: The proportion of accurate forecasts for positive outcomes relative to the total number of predicted positive outcomes.


TP÷(TP+FP)

Recall: The recall (or sensitivity) is the ratio of correctly predicted positive observations to all actual positives.


TP÷(TP+FN)

F1 Score: The F-1 Score is the harmonic mean of Precision and Recall, and is formulated as

(2×PRecision×Recall)÷(Precision+Recall)

F-0.5 and F-2 Scores: The F-β score is a generalization of the F-1 score, where *β* determines the weight of recall in the combined metric:

$$\left((1+\beta^{2})\times Precision\times Recall)÷((\beta^{2}\times Precision)+Recall\right)$$

Both false positives and false negatives in COVID-19 detection using X-ray images can have serious consequences. A false positive may result in unnecessary treatment, while a false negative may lead to a lack of necessary care. Therefore, a measure that considers both Precision and Recall, such as F-1 score, is often preferred. Choosing F-0.5 would prioritize Precision over Recall, potentially overlooking actual positive cases. F-2 prioritizes recall, potentially leading to more false positives. The authors likely selected the F-1 score owing to the specific demands and trade-offs of the task, where both types of errors are significant and a balanced approach is desired.

### 4.3 Experimental environment and computational complexity

The experiments were conducted in a controlled environment to guarantee the dependability and repeatability of the outcomes. The following are the crucial specifications of the hardware and software employed in the experiments:

Hardware Configuration:

Processor: Intel Xeon CPU with multiple cores to support parallel processing.

RAM: Sufficient memory to handle large-scale data.

GPU: High-performance Graphics Processing Units for accelerating deep learning computations.

Software Configuration:

Framework: Apache Spark, conducive to distributed computing.

Deep Learning Libraries: TensorFlow, PyTorch.

Programming Language Python is suitable for machine learning.

The controlled setting ensured that the experiments were conducted under uniform conditions, thereby eliminating potential discrepancies and biases.

#### 4.3.1 Computational complexity

The computational complexity of the model is crucial because it pertains to the efficiency and scalability of the algorithm. This can be examined through time and space complexities.

Time Complexity:

Apache Spark’s parallel processing significantly reduces the overall computation time. The complexity of the convolutional neural network models used (such as DenseNet-121 and ResNet50) contributes to the overall time complexity, which can be further analyzed based on the specific architecture of the chosen networks.

Space Complexity:

The distributed nature of data in Spark leads to increased memory utilization. Handling 6,500 images scaled to 235 × 235 pixels contributes to space complexity. The computational complexity of the proposed model strikes a balance between robust performance in COVID-19 detection using chest X-ray images and efficiency in terms of time and space. The selection of tools and techniques, including the Apache Spark framework and deep learning models, was tailored to meet the computational requirements of the task. Future work may focus on optimizing complexity to enhance the scalability and efficiency of the system.

### 4.4 Parameters selection for deep learning models

#### 4.4.1 Selection criteria

The systematic selection of hyperparameters for deep learning models, including DenseNet-121, ResNet50, ResNet18, and SqueezeNet, was conducted with careful consideration of primary factors such as performance and computational efficiency.

Performance Metrics: The hyperparameters were adjusted to achieve the best performance in terms of accuracy, precision, recall, and F1-score for COVID-19 detection.

Computational Efficiency: The parameter selection targeted a balance between model complexity and computational resources, such as processing time and memory usage.

Generalization Ability: To prevent overfitting, the hyperparameters were chosen to promote the model’s ability to generalize effectively to unobserved data.

Empirical Analysis: Based on prior empirical studies, the literature, and proven effectiveness in similar tasks, parameters were also selected.

#### 4.4.2 Specific parameters

Learning Rate: This parameter determines the size of the increment in the gradient descent process. It was selected through a search over a range of values using a grid search to determine the learning rate that minimized the loss function.

Batch Size: The number of training examples in one forward/backward pass was determined to strike a balance between the training speed and convergence stability, with the optimal batch size being selected.

Epochs: The number of complete passes through the training dataset was determined based on the observations of convergence patterns during training.

Activation Functions: The rectified linear unit (ReLU) activation function was selected for its ability to address the vanishing gradient issue and promote faster convergence.

Regularization Techniques: To avoid overfitting, dropout and L2 regularization were applied.

#### 4.4.3 Tools and techniques

Grid Search: A thorough search over a predetermined hyperparameter grid was performed to determine the optimal combination of parameters.

Cross-validation: To ensure reliable and robust hyperparameter selection, k-fold cross-validation was performed.

#### 4.4.4 Justification for utilising apache spark

The decision to use Apache Spark to process a large dataset of 6,500 images was driven by its ability to perform parallel and distributed computing. This allows efficient hyperparameter tuning by utilizing the parallel processing power of the system. With a large dataset, Apache Spark’s parallel processing capability enables faster experimentation, more effective tuning of the model, and ultimately, better performance.

Finally, the careful selection of parameters was a crucial step in constructing the deep learning models and was performed with meticulous attention to ensure the effectiveness, efficiency, and dependability of the proposed system.

### 4.5 Hyperparameter, overfitting, and model tuning

We have undertaken an extensive hyperparameter optimization process for our ensemble learning approach, amalgamating intricate architectures, such as VGG-16, VGG-19, and ResNet-50. Prior to integrating these models into our ensemble setup, we individually fine-tuned each model. Specifically, for the VGG-16, VGG-19, and ResNet-50 models, we meticulously adjusted crucial hyperparameters, including the learning rate, batch size, and weight decay, to ensure optimal standalone performance. Furthermore, recognizing the widespread application of VGG and ResNet architectures in image-processing tasks, we incorporated data augmentation techniques. This not only enhances the robustness of the models but also aids in improving generalization by exposing the models to diverse variations in the training data.

The following model tuning was performed. Prior to integrating these models into our ensemble setup, we individually fine-tuned each model. Specifically, for the VGG-16, VGG-19, and ResNet-50 models, we meticulously adjusted crucial hyperparameters, including the learning rate, batch size, and weight decay, to ensure optimal standalone performance.

## 5 Results

The datasets for multilevel classification to detect COVID-19 patients were acquired from Kaggle [46]. We collected two Datasets from the Kaggle repository. Dataset-1 had three categories of images: Normal, COVID-19, and Pneumonia. Dataset-2 contained only two types of images that were proven to be tuberculosis and normal. By combining these two datasets, 15, 819 images were obtained. The numbers of X-ray images of COVID-19, Normal Patients, Pneumonia, and Tuberculosis were 3616, 10,192, 1345, and 666, respectively. Fig 3 shows the sample dataset. The training phase used 75% of the dataset, whereas the testing phase used only 25%. The implementation used Python, Apache Spark, and machine-learning libraries. Apache Spark is utilized with MLlib of Apache Spark. Python programming language was used to train and evaluate the suggested pre-trained model using the Pyspark library of Apache Spark. All tests were conducted on Google Colaboratory utilizing a GPU graphic card and a Windows 10 operating system. Using the Adam optimizer, the CNN pre-trained models ResNet50, VGG-19, and VGG-50 were trained with initialization weights. All the experiments had the same batch size, learning rate, and number of epochs. After obtaining the results of these two models, the final step is to apply their outputs to the ensemble technique, that is, the Bucket of Model.

**Fig 3:** Sample of COVID-19, normal, pneumonia, tuberculosis.

The results of the model using cross-validation of the training and model evaluation with retrained embedding are presented in Table 1. The accuracy percentage of entity extraction was 88%, whereas that of intent was 74%. The pre-trained pipeline classified the purpose much better than extracting the entity because the intent classification had more than a 76% rate in F1-score and precision. However, removing the entity had a relatively low F1-score and precision of 52% and 72%, respectively. Our model had eight intents and more than 100 user examples. The overall accuracy of the defined intent was 75%, and the precision, recall, and f1-score were greater than 60%.

**Table 1:** CV pre-trained pipeline (test data).

Result	Intent Classification	Entity Extraction
Accuracy	74.8%	87.5%
F1-score	73.2%	48.5%
Precision	75.6%	69.3%

The supervised pipeline performed better in terms of intent classification based on precision (81%). In comparison, entity extraction had a higher accuracy rate of 87%, and intent classification had a good f1-score compared to entity extraction. This means that a supervised embedding pipeline works very well in classifying intent. The accuracy percentages of the models were 80.7%, 77.1%, 69.6%, and F1-score 72.1%, respectively as shown in Table 2.

**Table 2:** Supervised pipeline (test data).

Result	Intent Classification	Entity Extraction
Accuracy	80.7%	87.8%
F1-score	79.1%	51.1%
Precision	81.1%	67.5%

Fig 4 shows the improved accuracy of the training and validation. The improved results in the validation and training were due to an increase in epochs (e.g., 300). Similarly, Fig 5 shows the loss of training and validation, with minimal loss.

**Fig 4:** Model accuracy.

**Fig 5:** Model loss.

Further evaluation of the proposed system concerns the confusion matrix performance measures. The ML methods with ensemble approaches are VGG-16, VGG-19, and ResNet-50. The accuracies of all the techniques are shown in Figs 5 and 6. The precise values of accuracy for each model are also presented in Table 3. The precision, recall, and F-1 scores of the models are highlighted in Table 4. The training and testing errors are presented in Tables 5 and 6, respectively.

**Fig 6:** Performance of different models.

**Table 3:** Performance analysis.

DL Models	Accuracy
VGG-16	88.77
VGG-19	89.51
ResNet-50	90.90
Proposed Ensemble	94.31

**Table 4:** Precision, Recall, F1 Score.

Model	Values			
VGG-16		**Precision**	**Recall**	**F1-Score**
	**0**	0.88	0.97	0.94
	**1**	0.6	0.15	0.23
VGG-19		**Precision**	**Recall**	**F1-Score**
	**0**	0.89	0.98	0.95
	**1**	0.5	0.01	0.01
ResNet-50		**Precision**	**Recall**	**F1-Score**
	**0**	0.91	0.98	0.95
	**1**	0.61	0.4	0.5
Proposed Ensemble		**Precision**	**Recall**	**F1-Score**
	**0**	0.93	0.99	0.97
	**1**	0.79	0.51	0.67

**Table 5:** Training error.

Model	Training Error
VGG-16	0.20667
VGG-19	0.09968
ResNet-50	0.00034
Proposed Ensemble	0.00027

**Table 6:** Testing error.

Model	Testing Error
VGG-16	0.19989
VGG-19	0.12921
ResNet-50	0.07438
Proposed Ensemble	0.04547

Table 3 presents an overview of the accuracy metrics for the different Deep Learning (DL) models under consideration: VGG-16, VGG-19, ResNet-50, and our proposed Ensemble model. As demonstrated, the proposed Ensemble model boasts an accuracy rate of 94.31%, which surpasses other standard models. Specifically, this represents an improvement of approximately 3.41% over the closest competitor, ResNet-50, which has an accuracy rate of 90.90%.

Table 4 provides an exhaustive insight into the precision, recall, and F1-score metrics of each model for two classes: class 0 and class 1. It is evident that the proposed Ensemble model outperforms in nearly all metrics, especially in the F1-score and precision for class 0. These metrics are particularly crucial for medical applications where false positives and false negatives can have serious consequences. The proposed model presents a balanced compromise between precision and recall, as reflected in the F1-Score of 0.97 for class 0 and 0.67 for class 1.

Tables 5 and 6 focus on the error rates during the training and testing phases for each model. Significantly, our proposed Ensemble model exhibits the lowest training error of 0.00027 and testing error of 0.04547. This low level of error indicates that the model is not only able to learn the features efficiently but is also highly effective when generalising to unseen data. Compared to the ResNet-50 model, which has a training error of 0.00034 and a testing error of 0.07438, the proposed Ensemble model shows marked improvements.

## 6 Conclusions

The outbreak of COVID-19 has caused a global health crisis that requires the early detection and diagnosis of effective containment and treatment. Current methods for COVID-19 detection have limitations and there is a need for innovative solutions. This article proposes a novel architecture for detecting COVID-19 from chest X-ray images using data science and machine-learning techniques. This architecture uses a parallel and distributed framework, ensemble learning methods, and authentic real-time data from Pakistan to improve the accuracy of the detection process. The results demonstrate the effectiveness of the proposed architecture, offering a significant contribution to the current tools and techniques for COVID-19 detection using medical imaging. This study also identifies limitations and provides a path for future research. This study aimed to address the crucial challenge of identifying COVID-19 from chest X-ray images using cutting-edge data science and machine learning methods. The proposed architecture utilizes a parallel and distributed framework that incorporates ensemble learning techniques to accelerate both training and execution times. The approach was tested using genuine and reliable real-time data, including a comparison with state-of-the-art models, which confirmed its effectiveness.

### 6.1 Limitations

Despite these promising results, this study has some limitations that should be acknowledged. While the parallel and distributed frameworks improve training efficiency, they may also introduce complexity and require significant computational resources. Additionally, the choice of models and their ensembles may introduce bias, affecting the model’s ability to generalize. Finally, the evaluation of the model against state-of-the-art models may be limited by the scope and design of the comparative evaluations.

### 6.2 Future scope

Recognizing these limitations provides opportunities for future research, such as investigating the model’s performance across diverse datasets and demographics to enhance its generalizability. Other areas of investigation include reducing computational requirements without compromising the accuracy or training time, exploring more advanced ensemble techniques to reduce bias and improve robustness, and conducting a more comprehensive comparison with existing models using various performance metrics to offer a more complete evaluation.

The proposed architecture represents a valuable addition to the field of COVID-19 detection from chest X-rays, with notable improvements in both training and execution times. However, some limitations indicate the need for further refinement and exploration. The delineated future scope presents a clear path for subsequent research endeavors, underscoring the significance and potential impact of this work within both the scientific community and broader healthcare landscape.
